The article "The Efficacy of Remifentanil Combined with Propofol in Craniotomy for Tumor Was Evaluated by Wake Quality, Hemodynamics, and Adverse Reactions" was retracted in 2023. Reasons: unreliable results or conclusions; lack of ethics approval or compliance; concerns about the data; concerns about the peer review.

# The Efficacy of Remifentanil Combined with Propofol in Craniotomy for Tumor Was Evaluated by Wake Quality, Hemodynamics, and Adverse Reactions

**DOI:** 10.1155/2022/4861043

**Published:** 2022-07-18

**Authors:** Qiang Zhou, Yanan Han, Jun Chen

**Affiliations:** ^1^Department of Anesthesiology, Tianjin Huanhu Hospital, Tianjin 300350, China; ^2^Department of Operation Room, Tianjin Huanhu Hospital, Tianjin 300350, China

## Abstract

In order to investigate the effect of remifentanil combined with propofol on awakening of craniotomy for tumor, a retrospective analysis is conducted. 86 patients who underwent craniotomy for brain tumor in our hospital from July 2020 to December 2021 are chosen to observe the quality of awakening, hemodynamic parameters, and the occurrence of adverse reactions. All patients are divided into group A (*n* = 43) and group B (*n* = 43) according to the use of anesthesia drugs. The intraoperative awakening quality and the hemodynamic parameters during different periods of the two groups are compared. The experimental results show that the incidence of postoperative adverse reactions in group B is significantly lower than that in group A (*P* < 0.05). It is clearly evident that remifentanil combined with protocol has good intraoperative wake-up effect in craniotomy for tumor and maintain the hemodynamic stability of patients. Also, it can obtain high wake-up quality and effectively reduce postoperative adverse reactions.

## 1. Introduction

As a kind of skull surgery, surgery is often used to treat various brain diseases, such as cerebral hemorrhage, intracranial tumors, and ventriculoperitoneal shunt. In craniotomy for craniocerebral tumors, the patients with different tumor locations are likely to cause neurological damage in the adjacent areas [1]. It will lead to further language or motor dysfunction after surgery. Moreover, the prognosis of these patients is seriously affected, and their quality of life is reduced [2]. Therefore, how to remove tumors to the maximum extent under the premise of ensuring brain function is a common concern of surgeons. With the continuous development of medical technology, intraoperative arousal anesthesia technology has gradually appeared in people's vision [3]. It can ensure that patients remain awake during craniotomy, so as to help doctors determine the functional area of the brain and the scope of tumor resection. This is helpful to improve the accuracy of tumor resection during operation [4]. However, in clinical application, although this method can accurately remove brain tumors, it will cause serious physical stress response and postoperative complications. Therefore, the use of narcotic drugs during surgery is particularly important [5]. At present, the commonly used narcotic drugs in clinic include propofol, remifentanil, dexmedetomidine, and fentanyl. Their application effects in surgery have their own advantages, but there are relatively few studies on the combined use of intraoperative arousal technology [6]. This study retrospectively analyzed the clinical data of patients with craniocerebral tumors who underwent craniotomy in our hospital and compared the clinical efficacy of remifentanil combined with propofol in the implementation of intraoperative arousal technology. The research findings can provide corresponding theoretical basis for further improving the prognosis of such patients.

This paper is organized as follows: Section 2 discusses the related work.  Section 3 is our proposed awakening methods and wake up quality assessment.  Section 4 is the comparative analysis of experimental data and results. Finally, the work summary and future work of this paper are summarized in Section 5.

## 2. Related Work

Craniocerebral tumors, as tumors occurring in intracranial tissues or brain metastasis, are often clinically presented as increased intracranial pressure or other neurological symptoms, of which malignant tumors account for more than half. Currently, craniotomy is the main treatment for intracranial tumors in clinical practice [7, 8]. According to incomplete data statistics, the incidence of glioma among all intracranial tumors is about 80% of the primary intracranial malignant tumors, and the higher the classification of WHO central nervous system tumors, the higher the malignant degree of tumors, the more difficult the operation, and the worse the prognosis effect [9]. Other intracranial tumors included meningioma, acoustic neuroma, and brain metastases, have been reached on the unified conclusion about the pathogenesis, but most of the research have ionizing radiation was the cause of formation of meningioma, and glioma important risk factors for other risk factors include viral infections, such as allergic disease [10]. As an important treatment for intracranial tumors, craniotomy is faced with the main problem of precise localization and resection of lesions while avoiding neurological impairment, and intraoperative awakening technology provides technical support for solving this problem [11]. Therefore, this study is aimed at laying a theoretical foundation for improving the prognosis of patients undergoing craniotomy for tumor and improving the surgical effect by exploring the specific efficacy of different anesthetic drugs in the development of intraoperative awakening.

Some research results suggest that fentanyl propofol combined anesthesia has a higher effect of intraoperative resuscitation. It can effectively make the patients have relatively clear consciousness after awakening and can carry out activities according to instructions [12, 13]. In addition to the hemodynamic parameters observed at different times during the operation, the hemodynamic society of patients changed to a certain extent with the progress of recovery during the operation. It is necessary to verify the role of fentanyl combined with propofol in maintaining the stability of vital signs during operation. Some studies have shown that fentanyl, as an opioid stimulant, enters the body in a balanced blood brain for about 1 minute and is rapidly hydrolyzed by tissue and blood. Therefore, it has rapid analgesic effect, short elimination half-life, end-stage half-life, and biological half-life of about 3 ~ 10 minutes. However, patients are easily affected by the side effects of naloxone. Therefore, postoperative nausea, vomiting, bradycardia, and other adverse reactions are easy to occur [14, 15]. However, propofol, as a short-acting intravenous anesthetics of the venomal class, can be distributed throughout the body about 40 s after intravenous injection and make patients quickly fall into sleep state. Moreover, it can inhibit throat reflex to some extent and effectively reduce postoperative adverse reactions such as intraoperative nausea, vomiting, and irritability [16, 17]. So the two drugs used in combination can not only achieve relatively fast and stable intraoperative anesthetic effect, and the combination of propofol use can reduce the dosage of fentanyl, thereby reducing respiratory effects produced by rui fentanyl, and inhibition of intraoperatie injury stimulation, thus maintaining intraoperative hemodynamic stability, consistent with the findings [18]. In addition, OAA/S score was also used to compare the sedation degree of patients in the two groups during awakening. Therefore, it is necessary to further provide a solid foundation for intraoperative focus localization and tumor resection to improve the postoperative prognosis [19, 20].

## 3. Our Proposed Awakening Methods and Wake Up Quality Assessment

A retrospective analysis was performed on 86 patients who underwent craniotomy for brain tumor in our hospital from July 2020 to December 2021. All subjects received intraoperative wake-up anesthesia and were divided into group A (*n* = 43) and group B (*n* = 43) according to the use of anesthesia drugs. The comparison of baseline data between the two groups is shown in Table 1. All patients included in the study signed informed consent before surgery and obtained the right to know and consent to the intraoperative operation. Clinical data and general information obtained in this study are kept confidential and will not be used for other purposes.

Patients are included according to the following criteria: (1) they met the specific clinical criteria of craniotomy for craniocerebral tumors, (2) complete clinical data and general information, (3) sign informed consent before operation, (4) high treatment compliance and coordination ability, and (5) ASA class I ~ II. In addition, the exclusion criteria are as follows: (1) accompanied by mental illness; (2) patients with a history of allergy to narcotic drugs during operation; (3) patients whose physical condition cannot tolerate the operation; (4) patients with coagulation function or congenital immune dysfunction; and (5) complicated with heart, liver, kidney, and other major organ diseases.

### 3.1. Intraoperative Anesthesia and Awakening Methods

Patients in both groups received preoperative training to fully understand intraoperative operations and related events, and routine ECG monitoring was established after entering the operating room to monitor arterial pressure, heart rate, oxygen saturation, and other hemodynamic parameters in real time.

In group B, fentanyl, rocuronium, and propofol were used for rapid induction, then laryngeal mask was placed, and scalp nerve block was performed with ropivacaine hydrochloride. Propofol was injected with 0.8 mg·kg^−1^·H^−1^ and remifentanil with 0.8ug·kg^−1^·min^−1^; BIS value was maintained at 40~50 during the operation; after the removal of bone flap, 1-2% lidocaine was given to cover the epidural according to different conditions of each patient; infiltration anesthesia was performed for 20 minutes. Pump infusion of propofol and remifentanil was gradually stopped 20 min before awakening. Patients were awakened with gradual recovery of respiration, SPO_2_ ≥ 98%, PetCO_2_ at 35-45 mmHg, and BIS at 75-80. Patients were required to perform body movements and verbal commands, and changes in hemodynamic parameters were observed. Remifentanil and propofol were repumped at the end of the functional area surgery to maintain BIS at 60 hours and maintain spontaneous breathing until the end of the surgery. Patients in group A underwent the same operation as those in group B, and only remifentanil was used for anesthesia.

### 3.2. Wake Up Quality Assessment

This method is used to evaluate the degree of wakefulness of patients during awakening, which is divided into grades I ~ IV. Level I means that patients have clear consciousness after awakening and can carry out activities according to instructions. Level II means patients can barely open their eyes after calling, but cannot move their limbs as instructed. Grade III is sudden awakening, accompanied by restlessness of limbs. Grade IV is sudden awakening with severe limb agitation.

### 3.3. Alertness and Sedation Score

The scale is mainly used to evaluate the degree of sedation of patients during intraoperative awakening. The scale is mainly evaluated from four aspects, including reaction, speech, facial expression, and eyes/eyes. The score range is 1-5, and the higher the score is, the clearer the patient's consciousness and the higher the degree of sedation.

### 3.4. Technical Roadmap

As shown in Figure 1, the technical roadmap illustrated the specific research steps to investigate the effect of remifentanil combined with propofol on awakening of craniotomy for tumor. All subjects received intraoperative wake-up anesthesia and are divided into group A (*n* = 43) and group B (*n* = 43) according to the use of anesthesia drugs. Group A is given remifentanil. Group B is combined with propofol on the basis of group A, and the intraoperative awakening quality of the two groups will be compared. The hemodynamic parameters of the two groups are compared before anesthesia (*T*1), 10 min before awakening (*T*2), during awakening (*T*3), and 10 min after awakening (*T*4). Improved alertness and sedation score (OAA/S) are used to compare the sedation degree between the two groups during awakening. The incidence of postoperative adverse reactions is compared between the two groups.

## 4. Comparative Analysis of Experimental Data and Results

### 4.1. Comparison of Intraoperative Awakening Quality

Results of intraoperative awakening quality showed that the number of patients with grade I awakening quality in group B was significantly higher than that in group A (*P* < 0.05). Although there was no significant difference in other awakening quality grades (*P* > 0.05), the number of patients with grades III and IV in group B was lower than that in group A, as shown in Table 2. The results of the evaluation of arousal quality in this study showed that the intraoperative arousal quality of group B was grade I significantly higher than that of group A, and there was no difference in the classification of other cases, but the arousal quality of group B was grade III ~ IV lower than that of group A.

### 4.2. Changes in Intraoperative Hemodynamic Parameters

Change of MAP is illustrated in Table 3 and Figure 2. In Table 3, “a” means that compared with *T*1, a*P* < 0.05, “b” represents b*P* < 0.05 compared with *T*2, “c” indicates that compared with *T*3, c*P* < 0.05, and “d” represents d*P* < 0.05 compared with *T*4. In Figure 2, “a, b, c” means that if the same letter is shared between groups, respectively. “#” indicates that *P* < 0.05 between the two groups compared at the same point. Besides, change of HR can be observed in Table 4 and Figure 3.  Table 5 and Figure 4 show the change of SPO_2_ at each time point. No significant differences were found in hemodynamic parameters of the two groups at stage *T*1 and *T*2. With intraoperative awakening, MAP and HR increased in both groups, while SPO_2_ decreased. However, the range of change in group B at *T*3 and *T*4 was significantly lower than that in group A (*P* < 0.05).

### 4.3. The Degree of Sedation during Intraoperative Awakening in Both Groups

The sedation degree of group B during awakening was significantly higher than that of group A (*P* < 0.05), as shown in Table 6.

### 4.4. The Incidence of Postoperative Adverse Reactions

The incidence of postoperative adverse reactions in group B was significantly lower than that in group A (*P* < 0.05), as shown in Table 7.

Through the above experimental results, it can be observed that the incidence of postoperative adverse reactions in group B is significantly lower than that in group A (*P* < 0.05). It is clearly evident that remifentanil combined with protocol has good intraoperative wake-up effect in craniotomy for tumor and maintain the hemodynamic stability of patients. Also, it can obtain high wake-up quality and effectively reduce postoperative adverse reactions.

## 5. Conclusions and the Future Work

In this study, a retrospective analysis is conducted to investigate the effect of remifentanil combined with propofol on awakening of craniotomy for tumor. From the experimental results, it can be observed that red fentanyl combined propofol in the intraoperative wake can significantly improve the quality of wake up and keep the patients with stable hemodynamic parameters in the process of operation. It can obtain high sedation during wakes up and avoid patients with relatively strong stress response to environmental stimuli, which influence the result of the surgery. In addition, remifentanil combined with propofol can effectively reduce the incidence of postoperative adverse reactions and has high clinical value in improving postoperative prognosis. However, due to the limited number of samples, the study also has certain limitations, and the accuracy of the study results needs to be further discussed. For the future work in this paper, we will expand the number of patient samples in the following research and examine various stress response indicators to further explore the specific efficacy of remifentanil combined with propofol in the intraoperative wake-up technology.

## Figures and Tables

**Figure 1:** Technology roadmap.

**Figure 2:** Change of MAP.

**Figure 3:** Change of heart rate.

**Figure 4:** Change of SPO_2_.

**Table 1:** The baseline data.

	A group (*n* = 43)	B group (*n* = 43)	*t*/*x*^2^	*P*
Age (years)	43.45 ± 5.21	44.08 ± 4.96	0.574	0.567
Gender			0.186	0.666
Man	22 (51.16%)	20 (46.51%)		
Woman	21 (48.84%)	23 (53.49%)		
BMI (kg/m^2^)	23.21 ± 1.89	23.18 ± 2.05	0.071	0.944
Level of education			0.162	0.482
Primary and below	11 (25.58%)	9 (20.93%)		
Junior to Senior High	24 (55.81%)	26 (60.47%)		
University and above	8 (18.60%)	8 (18.60%)		

**Table 2:** Comparison of intraoperative arousal quality.

Group	*n*	I	II	III	IV
A group	43	6 (13.95%)	13 (30.23%)	18 (41.86%)	6 (13.95%)
B group	43	14 (32.56%)	11 (25.58%)	12 (27.91%)	2 (4.65%)
*x* ^2^		4.170	0.231	1.843	2.205
*P*		0.041	0.631	0.175	0.138

**Table 3:** Change of MAP.

Group	*n*	*T*1	*T*2	*T*3	*T*4	*F*	*P*
A group	43	10.48 ± 1.36^cd^	10.29 ± 1.57^cd^	11.97 ± 1.72^abd^	12.64 ± 1.54^abc^	3.517	0.002
B group	43	10.45 ± 1.32^cd^	10.34 ± 1.54^cd^	11.14 ± 1.63^abd^	11.58 ± 1.48^abc^	3.295	0.025
*t*		0.104	-0.149	2.297	3.254		
*P*		0.918	0.882	0.024	0.002		

**Table 4:** Change of heart rate.

Group	*n*	*T*1	*T*2	*T*3	*T*4	*F*	*P*
A group	43	82.17 ± 7.74^cd^	80.88 ± 7.39^cd^	95.42 ± 8.49^abd^	98.41 ± 7.39^abd^	4.319	<0.001
B group	43	81.37 ± 7.59^cd^	80.58 ± 7.52^cd^	86.43 ± 7.84^abd^	89.38 ± 8.03^abd^	4.742	<0.001
*t*		0.484	0.187	5.101	5.426		
*P*		0.630	0.852	<0.001	<0.001		

**Table 5:** Change of SPO_2_.

Group	*n*	*T*1	*T*2	*T*3	*T*4	*F*	*P*
A group	43	99.21 ± 0.58^cd^	99.11 ± 0.61^cd^	97.12 ± 0.87^ab^	97.01 ± 0.63^ab^	2.102	0.182
B group	43	99.19 ± 0.60^cd^	99.09 ± 0.52^cd^	98.26 ± 0.76^ab^	98.02 ± 0.58^ab^	2.252	0.063
*t*		0.157	0.164	-6.471	-7.734		
*P*		0.875	0.870	<0.001	<0.001		

**Table 6:** OAA/S score comparison.

Group	*n*	OAA/S
A group	43	2.42 ± 0.59
B group	43	3.17 ± 0.64
*t*		-5.650
*P*		<0.001

**Table 7:** Adverse reaction comparison.

Group	*n*	Bradycardia	Restlessness	Nausea and vomiting	High blood pressure	Total number
A group	43	2	4	6	4	16 (37.21%)
B group	43	1	1	3	2	7 (16.28%)
*x* ^2^						4.807
*P*						0.028

## Data Availability

The simulation experiment data used to support the findings of this study are available from the corresponding author upon request.
